The article "Design and Analysis of a Low-Cost Electronically Controlled Mobile Ventilator, Incorporating Mechanized AMBU Bag, for Patients during COVID-19 Pandemic" was published in 2022. Journal: J Healthc Eng.

# Design and Analysis of a Low-Cost Electronically Controlled Mobile Ventilator, Incorporating Mechanized AMBU Bag, for Patients during COVID-19 Pandemic

**DOI:** 10.1155/2022/6436818

**Published:** 2022-03-30

**Authors:** Rohan Lal Kshetry, Arnab Gupta, Somnath Chattopadhyaya, Madhulika Srivastava, Shubham Sharma, Jujhar Singh, Anirban Das Gupta, S. Rajkumar

**Affiliations:** ^1^School of Nuclear Studies and Application, Jadavpur University, Kolkata 700032, India; ^2^Department of Mechanical Engineering, Indian Institute of Technology, Madras, Tamil Nadu, India; ^3^Department of Mechanical Engineering, Indian Institute of Technology (Indian School of Mines), Dhanbad 826004, India; ^4^Department of Mechanical Engineering, Amrita School of Engineering, Amrita Vishwa Vidhyapeetham, Chennai, Tamil Nadu, India; ^5^Mechanical Engineering Department, University Center for Research and Development, Chandigarh University, Mohali, Punjab, India; ^6^Department of Mechanical Engineering, IK Gujral Punjab Technical University, Kapurthala 144603, India; ^7^Department of Anatomy, AIIMS Kalyani, NH–34 Connector,Basantapur, Saguna, West Bengal 741245, India; ^8^Department of Mechanical Engineering, Faculty of Manufacturing, Institute of Technology, Hawassa University, Awasa, Ethiopia

## Abstract

The outbreak of novel COVID-19 has severely and unprecedentedly affected millions of people across the globe. The painful respiratory distress caused during this disease calls for external assistance to the victims in the form of ventilation. The most common types of artificial ventilating units available at the healthcare facilities and hospitals are exorbitantly expensive to manufacture, and their number is fairly inadequate even in the so-called developed countries to cater to the burning needs of an ever-increasing number of ailing human subjects. According to available reports, without the provision of ventilation, the novel COVID-19 patients are succumbing to their ailments in a huge number of cases. This colossal problem of the availability of ventilator units can be addressed to a great extent by readily producible and cost-effective ventilating units that can be used on those suffering patients during an acute emergency and in the absence of conventional expensive ventilators at hospitals and medical care units. This paper has made an attempt to design and simulate a simple, yet effective, mechanized ventilator unit, which can be conveniently assembled without a profuse skillset and operated to resuscitate an ailing human patient. The stepper motor-controlled kinematic linkage is designed to deliver the patient with a necessitated discharge of air at optimum oxygen saturation through the AMBU bag connected in a ventilation circuit. With the associated code on MATLAB, the motor control parameters such as angular displacement and speed are deduced according to the input patient conditions (age group, tidal volume, breathing rate, etc.) and thereafter fed to the controller that drives the stepper motor. With a proposed feedback loop, the real-time static and dynamic compliance, airway resistance values can be approximately determined from the pressure variation cycle and fed to the controller unit to adjust the tidal volume as and when necessary. The simplistic yet robust design not only renders easy manufacturability by conventional and rapid prototyping techniques like 3D printing at different scales but also makes the product easily portable with minimal handling difficulty. Keeping the motto of Health for All as envisioned by the WHO, this low-cost indigenously engineered ventilator will definitely help the poor and afflicted towards their right to health and will help the medical professionals buy some time to manage the patient with acute respiratory distress syndrome (ARDS) towards recovery. Moreover, this instrument mostly includes readily available functional units having standard specifications and can be considered as standard bought-out items.

The article "Design and Analysis of a Low-Cost Electronically Controlled Mobile Ventilator, Incorporating Mechanized AMBU Bag, for Patients during COVID-19 Pandemic" was published in 2022. Journal: J Healthc Eng.

## 1. Introduction

Mechanical ventilation, preferably used to provide an auxiliary flow of oxygen gas through the trachea or windpipe to the respiratory-challenging human subjects, is an issue of utmost importance in the current pandemic scenario of the world. It was mentioned in earlier days and since that period of time, methodologies and instrumentation applied have been evolving through continuous enhancements and augmentation. Claudius Galenus, a physician and surgeon of the Roman Empire, was among the initial researchers to emphasize state about the mechanical aspects of the ventilation process and its delicate relationship with the functioning of the lungs nearly 2,000 years before [1–5]. In Ayurveda (ancient Indian medical science), it is categorically stated that the functions of *prana vayu* are responsible for the process of respiration in the human body. The channels or tracts (*Srotas*) in which *prana vayu* flows are called *pranavaha srotas*. *Prana vayu* is compared with the atmospheric oxygen that was called *amlajan*, meaning the base constituents of acids is necessary to carry out the vital functions of life. The facts as described by ayurvedic scholars in earlier days in the Gupta period depict a clear and categorical feature mentioned in the process of respiration in human subjects [3, 6–13].

Later on, numerous researchers and scientists have sincerely made an attempt to comprehend and critically analyze this mechanism [3]. In the middle of the twentieth century, different one-directional valves got fabricated incorporating diverse intricate features to aid the process of respiration. Several varied manual ventilation methods were discussed and utilized, and two of them are mouth-to-mouth and mouth-to-nose models. Among them, the “bag-valve-mask” procedure was extensively popular and specifically used for emergencies with initial preemptive offline settings [4].

The article "Design and Analysis of a Low-Cost Electronically Controlled Mobile Ventilator, Incorporating Mechanized AMBU Bag, for Patients during COVID-19 Pandemic" was published in 2022. Journal: J Healthc Eng.

Mechanical ventilation assisted with typical bag valve mask is predominantly used procedures to deliver manually some positive pressure in the ventilation process to the human subjects suffering critically from respiratory ailments [11–18]. From the time period of mid-sixteenth century till the early twentieth century, specially fabricated ventilation techniques described in the contemporary literature refer only typical mouth to mouth modes of operation and the practice of using bellows [1, 19–33]. In fact, in the fifteenth century, Paulus Bagellardus, a professor of medicine at the University of Padua, reported the first known documents on neonatal ailments and discussed general mouth-to-mouth resuscitation aided by advising midwives to deliver oxygenated air pressure into the mouths of the newly born subjects if there is the possibility of the absence of respiratory activities [3, 5]. This occurrence manifested that mouth-to-mouth mode-based ventilation strategies were already in vogue at that period of time. In mid-sixteenth century, after further investigations on a porcine model, Andreas Vesalius, a Flemish anatomist and physician accorded, gave recommendations to deliver air pressure into the windpipe/trachea with the help of a typical reed for enhancing the survival rate of the animal. Matteo Realdo Colombo, a famous Italian professor of anatomy as well as a surgeon at the University of Padua, has been served as a successor for this traditional practice about a decade later. He also mentioned this tracheotomy (an incision in the windpipe made to relieve an obstruction to breathing) based methodology. After one century, Robert Hooke, a very reputed scientist of the seventeenth century having terrific acumen in experimentation, recreated the instrumental strategy of Vesalius utilizing the model of a strangled chicken, which was factually ventilated with the help of bellows. On the basis of his experimentation, Hooke revealed the fact that with the aid of this type of model that the leakage of the fresh air was the root cause of death [1] in a substantial number of human cases suffering from nontrivial respiratory ailments.

The article "Design and Analysis of a Low-Cost Electronically Controlled Mobile Ventilator, Incorporating Mechanized AMBU Bag, for Patients during COVID-19 Pandemic" was published in 2022. Journal: J Healthc Eng.

In the eighteenth century, mouth-to-mouth ventilation case was first conveyed for a coal miner. The resuscitation was performed by the surgeon William Fossach [6]. He presented the case of mouth-to-mouth rescue [7]. In the late eighteenth century, Baron Antoine Portal gave a proposition for typical cases related to respiratory disorders, to inflate the lungs of the neonatal subjects with air. The Scottish surgeon John Hunter (13 February 1728–16 October 1793) propagator of such instrumental strategies in medical treatment and finally arduously fabricated human bellows equipped with pressure relief valves. He subsequently gave recommendations to the Royal Human Society for the urgent requirement of using mechanical ventilation on an emergency basis for resuscitation [3, 7, 33]. In addition to that, he stated that in order to decrease inflation of the stomach mild pressing of the larynx against the vertebrae will be an effective strategy measure [2, 7]. Royal Human Society and the French Academy of Medicine rejected the strategy plan of the use of bellows for enhancing mechanical ventilation for inadequate safety measures. Later John Fothergill recommended unique advantages of the mouth-to-mouth-aided mechanical ventilation in comparison to the bellow assisted ventilation during resuscitation [3, 7]. He deliberated that the heat and moistened state of the breathing air would be more effective to enhance the air circulation in comparison to the traditional way of supplying the cold and chilling air out of a pair of bellows to the ailing human subject without incurring further injuries [2]. In fact, with mouth-to-mouth mechanical ventilation, it is not possible to upsurge pressure to a level that the human subject is capable of generating. A descent illustration of efficacious bellow-assisted mechanical ventilation has been appropriately emphasized by Fell in a reported clinical pilot study [1]. Brain and Galen emphasized stressed the requirement for initial use of the bellows and prescribed a typical graduated bellows depending on the size of the human subject to decrease hyperventilation with greater volumes that probably can inflict additional injuries related to barotrauma [1]. In the mid-twentieth century, Peter Josef Safar vouched for the effectivity of mouth-to-mouth ventilation over other conventional procedures of typical manual ventilation in a brave and praiseworthy clinical trial  [10, 12, 33].

In 1950s, a different one-directional valve was fabricated with versatile features. The initial bag-valve-mask concept was evolved in the mid-twentieth century by the German doctor Holger Hesse and his partner, Danish physician Henning Ruben. They invented a nonelectric, self-inflating resuscitator. A typical terminology “Ambu” (artificial manual breathing unit) was used, and it was fabricated and sold in the markets in 1956 [9, 12, 33–42].

The article "Design and Analysis of a Low-Cost Electronically Controlled Mobile Ventilator, Incorporating Mechanized AMBU Bag, for Patients during COVID-19 Pandemic" was published in 2022. Journal: J Healthc Eng.

Although Hjelmgren et al. has discussed the incompatibility between the breathing system between the patient and the ventilators [43], they have emphasized the fact that mechanical ventilation has a comparatively longer cycle time in comparison to the natural breathing system of a human being. They have critically analyzed the cost-saving aspects of adaptive artificial ventilation systems. To minimize the asynchronous activities, they have proposed a system of adaptive adjustment through the recording of esophageal reading electrical responses through nasogastric channels. They have carried out a detailed comparison between neurally adjusted ventilatory assist controls with traditional pressure support ventilation [43]. The same has been analyzed by Raymond et al. who have deliberated about a scalable use of ventilators on an emergency basis with a special reference to the present COVID-19 crisis [44]. They have emphasized the fact of the current supply chain crisis of ventilators in the pandemic situation. They reported that most of the respiratory failure cases are due to the heterogeneous pulmonary parenchymal involvement in the pulmonary vascular injury. They have proposed a single-use low-cost ventilator designed and built in accordance with the emergency use international guidelines provided by competent international agencies of the USA where an external gas supply is maintained into the ventilator with some and time-controlled limited flow [44]. Moreover, Cole et al. have discussed an economically viable ventilator in the pretext of the COVID-19 pandemic situation where the constituent components will be easily available in the market at affordable cost with ample compatibilities with a robust capability of providing sufficient oxygenation and ventilation [45]. They have proposed a hybrid form of pneumatic type ventilator with various solenoid valves, a pressure chamber with an expiratory pressure valve and with suitable instrumentation for control. The specifications of the proposed ventilator are tidal volumes of 300–800 mL and positive end-expiratory pressure of 0–20 cm H_2_O. They have estimated a cost of US$ 250 for each ventilator for carrying out the rudimentary ventilation activities for the ailing patients [45]. Also, Swaroop et al. has made an attempt to examine presently available technologies for economically affordable transportable mechanical ventilators [46]. They have various strategies of fabricating low-cost ventilators, which incidentally have similar features to the traditional ventilators used in hospitals. The article elaborates the concept of the design and subsequent fabrication of a multiple-use, economically viable portable mechanical ventilator. The major feature of such ventilators is the sophisticated monitoring and control of the different major process parameters like tidal volume, breaths in a minute, the ratio of inspiration to expiration ratio, and last but not least the positive end-expiratory pressure. In the present perspective, these mechanical low-cost ventilators can be beneficial in reliable delivery of respiratory support to the COVID-19-infected subjects and similar precarious cases [46].

The article "Design and Analysis of a Low-Cost Electronically Controlled Mobile Ventilator, Incorporating Mechanized AMBU Bag, for Patients during COVID-19 Pandemic" was published in 2022. Journal: J Healthc Eng.

These mechanical ventilation units are undeniably necessary as respiratory support systems for ailing human subjects who encounter respiratory suffering resulting from any disease or ailment. It generally comprises intricate parts such as compressor, accumulator, different control valves, transmission lines, filters, actuator circuits, sensors, and a control console. All this incorporation imparts huge costs to the entire ventilator unit. Commercially available ones that are utilized in the hospitals range from $8,000 to $30,000 or sometimes even more (with various other add-on features). Consequentially, the number of such currently available machines is also not high. During the torrid times of pandemic-like situations, the novel COVID-19, or severe acute respiratory syndrome (SARS), that had occurred in the past in the world, has witnessed the exponential surge in the number of human subjects suffering from respiratory distress, thus calling for the urgent need of mechanical ventilation assistance. The inability to provide ventilator support to all the patients due to an inadequate number of ventilators available at the hospitals or ad hoc healthcare facilities has led to a huge number of casualties. The same is even visible at present due to COVID-19 outbreak. During such a period, the ventilators are expected to run incessantly continuously for days or weeks as required by the ailing patient. This reduces the reliability and longevity of the machine parts with successive operating cycles and calls for adequate maintenance. Most of the time, maintaining or repairing such malfunctioning or inoperative ventilation systems is a tedious and painstaking task for hospital management, healthcare administration, and staff employees. Therefore, it essentially demands expert support with additional expenses and loss of precious time for appropriate adequate medical treatment of the subjects.

A simpler form of ventilation support in case of emergencies is through manual resuscitation using artificial manual breathing unit (AMBU) bag or bag-valve-mask (BVM) as depicted in Figure 1. It comprises a self-inflating silicone or rubber bag that is manually compressed and released to deliver a fixed tidal volume of air to the patient's lungs either through a mask or through intubation (the process of inserting a tube, called an endotracheal tube). Manual operation is not often a convenient and preferred option for the healthcare staff or the person attending the patient during an emergency. Keeping all these factors in mind, a very simple, rudimentary, easy to operate, and reliable ventilation unit incorporating an AMBU bag was incepted. It can be easily assembled and disassembled by any healthcare personnel without any extensive prior knowledge and training about the conventional ventilator parts and their assembly. The user interface is also very easy and convenient to operate and monitor and can be made better with further development. Most of the standard parts are available at medical equipment stores. The mechanized linkages can be conveniently manufactured using CNC milling machines or by rapid prototyping techniques such as 3D printing and fitted with commercially available ball bearings at the rolling joints. The electronic parts can also be procured, and the circuit can be developed with ease.

The article "Design and Analysis of a Low-Cost Electronically Controlled Mobile Ventilator, Incorporating Mechanized AMBU Bag, for Patients during COVID-19 Pandemic" was published in 2022. Journal: J Healthc Eng.

## 2. Scope and Significance of the Work

Since 2019, the world has been negatively affected by a positive-stranded enveloped RNA virus with a death toll of nearly 50 lakhs because of ARDS, and it has earned the nomenclature of severe acute respiratory syndrome coronavirus-2 (SARS-CoV-2). Due to the obvious existence of ACE-2 functional receptor, which is found largely in pulmonary epithelial cells, the respiratory system has emerged as one of the most common battlegrounds for coronavirus infection. Pulmonary epithelial cells (type1, type 2, and club cells) are present in the respiratory zone of lungs, and they are dedicated to promoting the diffusion and secreting surfactant; the latter is responsible for increasing compliance of lung, thereby preventing alveolar collapse. An additional zone in the lungs is the conducting zone, which is characterized by pseudostratified ciliated columnar epithelium, cartilage discontinuous plates, and elastic fibres.

In 20% of the infected human subjects patients, the culprit virus, with the help of the host receptor ACE-2, enters the type 2 pneumocytes, thereby leading to the formation cascade of inflammatory mediators and chemoattractants known as “cytokine storm.” While doing so, the involved T lymphocytes get accumulated in the lung tissue, thereby leading to diffuse alveolar damage; this eventually culminates in an acute respiratory distress syndrome. The pathophysiology is depicted in Figure 2 [13]. Mechanical ventilation is one of the mainstays in managing ARDS and hence is an issue of utmost importance in the current pandemic scenario of the world.

The article "Design and Analysis of a Low-Cost Electronically Controlled Mobile Ventilator, Incorporating Mechanized AMBU Bag, for Patients during COVID-19 Pandemic" was published in 2022. Journal: J Healthc Eng.

Mechanization of AMBU bag unit has been pursued by many researchers across the world using various mechanisms such as cam-and-follower [47], slider-crank [49, 50], rack and pinion [51], dual-cam [54], and several complex kinematic and pneumatic systems [48, 52, 53] leading to a number of patents and effectivity analyses. In most of these mechanisms, the AMBU bag is subjected to nonuniform clamping force as being pressed between one moving clamp and one fixed clamp. Some comprise several intricate mechanical parts that pose difficulty in handling and maintenance. Also, the overall units are bulky and difficult for portability and maintenance. To overcome this, we propose a robust and compact mechanism for holding the AMBU bag and subjecting it to successive compression/relaxation while imparting equal clamping thrust from either side. We augmented to this a simple electronically operated closed-loop control strategy for delivering correct tidal volume and also monitoring the airway resistance in successive breathing cycles.

## 3. Methodology

This section elaborately elucidates the design of the kinematic linkage driving the AMBU operation, the electronics associated, and the controlling strategy with real-time monitoring of patient airway pressure.

### 3.1. Mechanization of the AMBU Bag

The mechanism was designed and simulated using Autodesk AUTOCAD and Autodesk INVENTOR to obtain the requisite kinematic and dynamic properties during its motion. The mechanism comprises a crank with two slots on either side of its center, as seen in Figure 3. Two pushrods with rotating-sliding elements capable of rolling along the two crank slots are installed. Each pushrod connects to a clamping arm. As the crank is given different degrees of rotation in a particular direction (clockwise or anticlockwise) by a coupled stepper motor, both the clamps simultaneously slide inwards or outwards on horizontal linear guide rails, as depicted in Figure 4. On placing an AMBU bag in between the clamps, the motion of the clamps imparts compression and relaxation on the self-inflating bag. The stepper motor operates according to the controller outputs and renders very precise relative linear displacement to the clamps, hence compressing/relaxing the AMBU bag by modulated volumes. Thus, it serves the purpose of mechanizing the otherwise manual job of resuscitation, with requisite accuracy.

### 3.2. Patient Circuit

The pneumatic circuit denoting the flow of air and oxygen mixture through the AMBU bag and other attached accessories has been depicted in Figures 5 and 6. The inlet and outlet valves of the AMBU bag are essentially one-way valves and are also known as fish-mouthed valves due to their typical shape. From the AMBU bag, the compressed air flows through a Venturi meter installed along the flow line. The Venturi meter facilitates airflow rate measurement and also pressure monitoring through the usage of two fluid pressure sensors MPX5010 (Figure 7). In Figure 5, the first pressure sensor reads differential air pressure between the entry and throat sections of the Venturi and a second pressure sensor in line reads the absolute air pressure flowing through the circuit.

The article "Design and Analysis of a Low-Cost Electronically Controlled Mobile Ventilator, Incorporating Mechanized AMBU Bag, for Patients during COVID-19 Pandemic" was published in 2022. Journal: J Healthc Eng.

The sensors are calibrated to measure within a set range as required in a ventilation air circuit. These sensors can sense both gauge pressure at a section along the flow line as well as differential pressure between two sections along the flow line and produce respective output voltage signals as per Figure 8. Using the difference in pressure at Sections 1 and 2, that is, (P1–P2) as illustrated in Figure 6, the volumetric airflow rate through the circuit can be determined by plugging the values in equation (1). Thus, it facilitates a cost-effective real-time monitoring of dynamic air pressure and volume flow rate along the breathing cycle of the patient.

From the Venturi meter, the air is flown through a breathing tube into the face mask (or intubated into the respiratory tract of the patient) as depicted in Figure 5. The mask comprises a one-way inlet valve and a one-way expiratory valve. Sometimes, during positive pressure mechanical ventilation, it becomes necessary to maintain a positive end-expiratory pressure (PEEP) at the end of the respiratory cycle as shown in Figure 9. This is achieved by fitting a PEEP valve at the expiratory port. It can be adjusted to discrete levels of PEEP.

(1) $$\begin{array}{c} \text{Volumetric air flow rate},\;\overset{ο}{V}=\;A2\;\times \sqrt{\frac{2}{\rho }\times \frac{\left(P1-P2\right)}{1-{\left(A2/A1\right)}^{2}}}. \end{array}$$

### 3.3. Control Unit

The actuation of the kinematic mechanism narrated in Section 3.1 is achieved using a bipolar, 10.2 kg-cm torque stepper motor with a 1.8° step angle (Model NEMA23). The motor is driven by a 4.0 A 42V TB6600 motor driver circuit (Model- RMCS 3758), controlled by an Arduino UNO microcontroller for the test phase. It operates based on an algorithm that takes parameters such as patient age group, tidal volume, respiratory rate, and ratio of inspiratory time to expiratory time as preliminary inputs and accordingly adjusts the stepper motor's starting position, degree of rotation, and angular speed during forward and backward stroke (enabling compression and expansion stages). The clamps can take three initial reference positions for three different AMBU bags commercially available for adult, pediatric, and neonatal patients, being preset in the control algorithm. Subsequently, according to the input tidal volume, the clamps will reciprocate with respect to the initial reference position. To simulate this operation with realistic perception, a code was written and compiled on MATLAB R2013a, the result of which is illustrated in Figure 12.

The article "Design and Analysis of a Low-Cost Electronically Controlled Mobile Ventilator, Incorporating Mechanized AMBU Bag, for Patients during COVID-19 Pandemic" was published in 2022. Journal: J Healthc Eng.

To run the real-time monitoring and feedback loop, the data from the MPX5010 sensors are acquired and analyzed, according to an algorithm coded using MATLAB R2013a. The air pressure-vs-time and volumetric flow rate (discharge) vs time plots are obtained from the sensor data collected at a specific sampling rate of 10 ms. From the pressure-vs-time plot, it fairly assimilates a typical graph illustrated in Figure 10; the peak inspiratory pressure (PIP), plateau pressure (PLP), positive end-expiratory pressure (PEEP), inspiratory time (T_insp_), and expiratory time (T_exp_) values are extracted for every successive breathing cycle [34]. From the volumetric flow rate (discharge) vs time plots, actual instantaneous tidal volume and minute volume (for *n*-th breathing cycle) are obtained through integrating $\;\overset{ο}{V}$ (discharge) over the inspiratory time period (from Texp of (*n *– 1)-th cycle to T_insp_ of *n*-th cycle) according to equations (2)–(4). Then the obtained values are used to evaluate the static compliance, dynamic compliance, and airway resistance in that cycle, using equations (5)–(7). In addition, the actual delivered tidal volume is compared with the desired tidal volume (initial input) to calculate a compensatory error value, which is fed to the controller to adjust the motor controller parameter settings and further AMBU bag compression if and when the compensatory error value exceeds the threshold value. This acts as a feedback loop for delivering the correct amount of air to the patient throughout the ventilation process. In case of substantial variation between the real and set values, the controller is able to adjust the compression stroke length by changing the degree of rotation of the stepper motor.

(2) $$\begin{array}{c} \text{Tidal volume},\text{VT }=\;\int_{T\;\exp|\left(n-1\right)}^{T\text{insp}|\left(n\right)}\;\overset{ο}{V}\text{d}t\left(\text{integrated over an inspiration cycle}\right), \end{array}$$

(3) $$\begin{array}{c} \text{minute volume},\text{VE }=\text{VT }\times \text{ respiratory rate}\left(\text{RR}\right), \end{array}$$

(4) $$\begin{array}{c} \text{total cycle time}\left(\text{TCT}\right)=\text{inspiratory time}\left({\text{T}}_{\text{insp}}\right)+\text{ expiratory time }\left({\text{T}}_{\text{exp}}\right)=\frac{1}{\text{RR}}. \end{array}$$

Lung compliance is another important ventilation parameter that needs to be closely monitored, as it has been found to have a significant correlation with the mortality of ARDS patients diagnosed with COVID-19 [35]. It is defined as the ratio of change in lung volume to the change in transpulmonary pressure. Transpulmonary pressure is the difference between the inside alveolar pressure and the outside pleural pressure. Normally, the total compliance of both the lungs is nearly 200 ml of air/cm of H_2_O for adults and, however, may vary significantly from patient to patient depending on the pathological conditions [36, 37]. Depending on whether there is any flow to the lungs and state of the muscles (relaxed or stretched) during measuring pulmonary compliance, it may be described as either static or dynamic. Static compliance represents the pulmonary compliance at a fixed volume when there is no airflow and the muscles are relaxed. This occurs when transpulmonary pressure is equal to the elastic recoil pressure of the lungs. Thus, it is a measure of only the elastic resistance. Dynamic compliance is measured during breathing and is used to monitor elastic resistance and airway resistance both [36]. Usually, pressure-vs-volume curves are used to depict the relationship between static and dynamic compliance whereby the slope of the curve denotes compliance [38]. Depending on the initial patient condition, limiting values of *X*_s_ and *X*_c_ can be set by the medical personnel, and in case of erratic deviation of the actual measured compliance, values from this range shall indicate worsening of patient condition, thereby necessitating immediate medical help.

(5) $$\begin{array}{c} \text{Static compliance }\left(X_{\text{s}}\right)=\;\frac{\text{VT}}{\;\left(\text{PLP }–\text{ PEEP}\right)}\frac{\text{mL}}{\text{cm }}\text{ of }{\text{H}}_{2}\text{O}, \end{array}$$

(6) $$\begin{array}{c} \text{dynamic compliance}\left(X_{\text{c}}\right)=\;\frac{\text{VT}}{\left(\text{PIP }–\text{ PEEP}\right)}\frac{\text{mL}}{\text{cm}}\text{ of }{\text{H}}_{2}\text{O}, \end{array}$$

(7) $$\begin{array}{c} {\text{R}}_{\text{aw}}\;=\;\frac{\left(\text{PIP }–\text{ PLP}\right)}{\overset{ο}{V}}\text{ cm of }\frac{{\text{H}}_{2}\text{O}}{\left(L/\text{sec}\right)}\;. \end{array}$$

Apart from the compliance parameters, the algorithm includes monitoring the airway resistance (R_aw_) determined from the real-time values of flow rate, PIP and PEEP read from the pressure variation curve on a respiratory time scale. The normal value of R_aw_ for an intubated and mechanically ventilated patient ranges from 5 to 10 cm H_2_O/L/sec [39]. The sudden surge in airway resistance caused by bronchospasm, mucus plug, excessive secretions, foreign body aspiration, or extrinsic airway compression is highly detrimental to the patient's ventilation and needs to be immediately addressed by the medical personnel. To include such a provision, an alarm is set to go off in case the airway resistance surpasses a preset limiting value.

The article "Design and Analysis of a Low-Cost Electronically Controlled Mobile Ventilator, Incorporating Mechanized AMBU Bag, for Patients during COVID-19 Pandemic" was published in 2022. Journal: J Healthc Eng.

## 4. Results and Discussion

The designed mechanism was simulated using Autodesk INVENTOR, and it performed suitably. The maximum and minimum interclamp distances for the chosen kinematic linkage are 16 cm and 1 cm, respectively, as depicted in Figure 11. However, the extreme (outward and inward) positions of the clamps are essentially different for different-sized AMBU bags, and the dimensions of the mechanism's links have been chosen to accommodate all the standard AMBU bags-adult, pediatric and neonatal, within the interclamp space. Overall, the actuation unit is compact and can be easily accommodated in a nominal volume space of 25 cm × 25 cm.

The stepper motor sets the starting position corresponding to the outmost clamp position as the reference. According to the initial set tidal volume and also the real-time deviation of actual delivered tidal volume in subsequent cycles (determined from the feedback loop compensation) within a specified tolerance of +/− 25 mL about the set tidal volume, the stepper motor decides the angle of rotation for every successive cycle. The angular speeds of the motor during the compression and relaxation strokes are set according to the input parameters: respiratory rate (breaths per minute) and expiratory time:inspiratory time (T_insp_:T_exp_) ratio, denoted by “*t*” in Figure 12.

After assembling and carefully putting the sterilized breathing mask on the patient, the ventilation controller is started. Figure 12 shows the initial parameters such as patient age group: adult, *t*: 3, breathing rate (breaths/min): 15 (typical for a normal adult), and tidal volume (desired, ml): 700 that are taken as a typical input during the initiation of AMBU bag ventilation unit from the attending personnel. Accordingly, the controller sets the initial starting position: ∼8.83° (with respect to a fixed origin), angle of rotation to impart compression stroke by clamps: ∼82.35° (with respect to starting position), motor angular speed during compression stroke (inspiration): ∼13.72 RPM, and motor angular speed during relaxation stroke (expiration): ∼4.57 RPM. The AMBU bag shall start operating on the patient with these parameters.

The article "Design and Analysis of a Low-Cost Electronically Controlled Mobile Ventilator, Incorporating Mechanized AMBU Bag, for Patients during COVID-19 Pandemic" was published in 2022. Journal: J Healthc Eng.

With the successive breathing cycles, the real-time airflow-rate-vs-time plot obtained from the sensor data is analyzed to deduce the actual delivered volumetric flow (actual tidal volume) as discussed in the previous section. Pressure-vs-time plot is analyzed to extract PIP, PLP, and PEEP values for every successive breathing cycle.  Figure 13 illustrates a sample test run of the code, wherein the extracted values are typically used to deduce various output parameters. In the first breathing cycle, a lower actual tidal volume is presumed (emulating a real-time situation), which through the feedback loop induces a change in stepper motor control parameters. This further adjusts the AMBU bag compression/expansion strokes and brings the actual delivered tidal volume closer to the initial input tidal volume for the patient, in the next cycle (second breathing cycle for instance, in this case). The code also determines the static and dynamic compliance and airway resistance values (Figure 13). The loop runs infinitely until the ventilator is stopped or reset due to any medical condition.

Here, an instrument of ventilation has been proposed with a strong emphasis on the affordability of the users. A modular design equipped with a reliable control algorithm (pertaining to preliminary/remote treatment) is adopted for the instrument to render better maintainability. The standard components are chosen that can be conveniently purchased from the medical and electronics stores. This instrument can be further modified to incorporate more precise control facilities to address different challenging pathological conditions. Because of the affordable cost, this instrument can be installed with reasonable expenses in small clinics or even households and can be utilized as preliminary medical support in case of emergency situations where the ailing patients require urgent respiratory assistance.

This mechanized ventilator mainly works on a controllable breathing mode, which is entirely set by the operator. There are numerous cases when it may be painful for the patient on ventilation as in those cases heavy sedation is done to provide relief to the ailing patients. Quite often, this may be worsened by conditions such as barotrauma whereby the diaphragm and intercostal muscles of the patient resist the inhalation (solely controlled by the machine in this case). A closely controlled peak pressure and positive end-expiratory pressure maintained at every breath cycle somewhat prevent atelectasis and barotrauma [40]. Hence patient-triggered ventilation assistance such as pressure-triggered (activated by a drop in air pressure in the trachea of the patient, which indicates the expansion of the thoracic cavity) or flow-triggered ventilation (whereby a flow sensor detects airflow to the lungs of the patient trying to breathe) are generally preferred in conventional ICUs [41, 42]. In these cases, the breathing sequences are triggered by the patient and do not essentially require sedation. But these intricacies make the ventilation machines exorbitantly expensive. Further research and development to impart low-cost solutions incorporating the same are in the pipeline.

The article "Design and Analysis of a Low-Cost Electronically Controlled Mobile Ventilator, Incorporating Mechanized AMBU Bag, for Patients during COVID-19 Pandemic" was published in 2022. Journal: J Healthc Eng.

The related work has been reported by DeBoer et al. has discussed the design and subsequent fabrication of economically affordable mechanical ventilators based on indigenously developed components [55]. The basic design of such a ventilator was to function in hospitals and as well as in difficult-to-access locations, having the capability of negotiating with different gas pressures and unreliable power supplies. They have investigated the various issues of the development of a respiratory support system with minimum hassles [55]. Similarly, Vasan et al. discussed the development and fabrication of a rudimentary, portable, and economically viable ventilator that can be hastily manufactured with ease [56]. The features of those ventilators may be pressure-controlled with a robust design. Those designs are validated with the use of certified test lungs extended period of time. As per the International norms, these designs are validated with the use of certified test lungs extended period of time [56]. Du Pasquier et al. discussed the work of a novel design of a ventilator of affordable cost on the basis of automatic compression of a resuscitator bag [48]. The device is made of widely available parts. The control process of the device is to give continuous mandatory ventilation (CMV) and spontaneous breathing assistance [48]. Also, Chatburn and Mireles-Cabodevila deliberated the method of interaction between the ventilator and the human subject [57]. They have reported that there are approximately 300 commercial names for the methods of ventilation. They have proposed a classification system appropriate for comparing those methods [57]. The related results have been found by the Calderón et al. who have also proposed that new methods of the economically viable portable ventilator are indispensable in the present state of Pandemic [58]. They have reported that a research group in Spain has indigenously developed such low-cost ventilators having the rudimentary features of the traditional ventilators. A different airbag resuscitator is proposed in that system. Sensors and appropriate display facilities are incorporated into the device. Experimental study confirms the sturdy character of those designed devices [58].

The article "Design and Analysis of a Low-Cost Electronically Controlled Mobile Ventilator, Incorporating Mechanized AMBU Bag, for Patients during COVID-19 Pandemic" was published in 2022. Journal: J Healthc Eng.

The same reports have been concluded by El-Hadj et al. has reported that the mechanical ventilator based on piston-cylinder is comparatively more favorable for the patient [59]. The article carried out a numerical analysis for reliably predicting the deliverables of a low-cost mechanical ventilator [59]. Also, Tran et al. has made an attempt to design, fabricate with a monitoring model, and to simulate a traditional mechanical ventilator with features of portability, bioinspired mechanism, finger-like actuator, and so on [60]. The same results have been revealed by Al Husseini et al. who discuss the design of an economically viable portable mechanical ventilator for the challenging environment of developing and underdeveloped regions of the world [61]. Their proposed model is using bag valve mask with the actuation through a cam in a mechanized way without human intervention. Tidal volumes are adjusted through user-friendly knobs. The arrangement of alarms is also incorporated in the proposed device [61]. Acho et al. showed the fabrication of an economically viable open-source mechanical ventilator [62]. The proposed design utilizes only the locally available spares for ease of fabrication. They have described a numerical method for monitoring the pulmonary condition of the human subject. The features of their design are precise pressure measurements and suitable alerts for clinicians [62]. Similarly, Jonas et al. discussed the asynchronous behavior between the human subject and the breaths from the mechanical ventilator [63]. They reported that neurally adjusted ventilatory decreases this asynchrony in comparison to traditional pressure support ventilation systems. The researchers have conducted a health economic assessment of neurally adjusted ventilatory compared with the traditional pressure support ventilation system [63].

Thus, with the provision of the requisite applications of artificial intelligence, internet of things, and predictive monitoring for diagnostics, the ailing patients of difficult-to-access regions can be remotely serviced in the presence of operators of rudimentary handling knowledge and experiences. For the hygienic part, this instrument can be easily assembled and disassembled for sterilization of the constituent components after use. Replacing parts as and when necessary is also very convenient. It shall consume very less power, can be battery-operated in regions subject to frequent power cuts, is tightly regulated, is reliable, can be operated for a long duration, and can be conveniently replaced. It shall be a convenient substitution to the conventional manually operated AMBU bag, which is often exhaustive for the attendant. Here, one attendant can monitor multiple patients under ventilation. It shall prove much useful in times of pandemic causing acute respiratory distress syndrome (ARDS) when there is a huge dearth of ventilators at hospitals. Taking into account the expenses involved in manufacturing and assembling the proposed mechanized ventilator, it is downright much less compared to those used presently. A typical experimental model involving the abovementioned parts and other miscellaneous accessories can be conveniently procured from the market or fabricated in a conventional CNC milling machine and shall cost within INR 20,000. Alternatively, a rapid prototyping machine if available can be used to directly print the parts in 3D. To enhance the performance and longevity of the integrated electronic systems for real scenario implementation, the expenses incurred will increase. However, with bulk fabrication and production, the unit cost will evidently come down.

The article "Design and Analysis of a Low-Cost Electronically Controlled Mobile Ventilator, Incorporating Mechanized AMBU Bag, for Patients during COVID-19 Pandemic" was published in 2022. Journal: J Healthc Eng.

## 5. Conclusions

The article has made an attempt to design and simulate an economically viable artificial ventilator for the ailing human subjects needing an external respiratory support system in the present pandemic situation worldwide. The researchers here have aimed to design and develop a cost-effective, simple, yet effectively mechanized ventilator unit, which can be assembled without much hassle and can be operated to resuscitate a patient in dire need. The robust kinematic linkage and a simple closed-loop monitoring strategy reliably elevate the performance of a stand-alone manually operated AMBU bag, thereby proving as an effective adaptable alternative. The components of this machine can be fabricated precisely with the help of conventional CNC machine tools or even by rapid prototyping techniques such as 3D printing as per the intended standards and scales. In addition to that, the equipment consists mostly of readily available functional units, which can be considered as standard bought-out items. This study precludes the dynamic aspects of the kinematic linkage such as loads associated with the sliding/rotating elements (friction, normal force, and inertial moments), which may play an indispensable role in choosing the stepper motor model. Consequently, the inaccuracies induced by thermal and tribological factors during the continuous running of the mechanism have not been considered and may be taken as a follow-up study on the proposed design. Also, the algorithm can be improvised to incorporate patient-triggered ventilation by augmenting sensory units along the airflow circuit that can monitor the actual breathing cycle of the patient and make the AMBU bag actuation complaint to that. Although this simple, less costly instrument cannot exactly replace the ventilators available in the present market at an exorbitant price and enabled with much-sophisticated instrumentation and control, surely, it can be installed in small clinics at places having restricted access to ventilators or during transit periods in ambulances to address acute respiratory distress of the patients. This low-cost ventilator will certainly help us tackle not only the COVID-19 pandemic but also ARDS consequent to other causes, thereby addressing the slogan by WHO of Health for All.

The article "Design and Analysis of a Low-Cost Electronically Controlled Mobile Ventilator, Incorporating Mechanized AMBU Bag, for Patients during COVID-19 Pandemic" was published in 2022. Journal: J Healthc Eng.

## Figures and Tables

**Figure 1:** AMBU bag and its accessories (source: https://litfl.com/bag-valve-mask-bvm-ventilation/).

**Figure 2:** Pathophysiology of ARDS in COVID-19 infection [13].

**Figure 3:** Kinematic mechanism model for compressing AMBU bag: (a) without AMBU bag and (b) with AMBU bag.

**Figure 4:** Extreme positions of the AMBU bag pressing clamps.

**Figure 5:** Schematic of the mechanized AMBU bag circuit implemented on a patient model with an augmented closed-loop (feedback) control strategy.

**Figure 6:** Venturi meter diagram (source: https://litfl.com/bag-valve-mask-bvm-ventilation/ and https://circuits4you.com/tag/mpx5010dp/).

**Figure 7:** (a) MPX5010 fluid pressure sensor and (b) MPX5010 pin configuration for differential pressure measurement (source: https://circuits4you.com/tag/mpx5010dp/).

**Figure 8:** Variation of output voltage with pressure for MPX5010 (source: https://circuits4you.com/tag/mpx5010dp/).

**Figure 9:** (a) Positive end-expiratory pressure (PEEP) valve and (b) PEEP valve with BVM (source: https://emcrit.org/).

**Figure 10:** Typical airway pressure variation with time (source: respiratory mechanics in mechanically ventilated patients [34]).

**Figure 11:** Simulation sequence (extreme positions) of clamp motion for adult AMBU bag.

**Figure 12:** Test run of the code on MATLAB R2013a for motor control during initiation (no feedback).

**Figure 13:** Test run for pressure monitoring and feedback loop to control tidal volume through subsequent breathing cycles.

## Data Availability

The data presented in this study are available on request from the corresponding author.

## Additional Points

The trial registration number is 60047 (West Bengal, Medical Council of India), and the issue date of registration is 13 September 2004, issued by the West Bengal Medical Council.
